# A Metadecomposition of Clinical Value Assessed Using aEEG in Severe Neonatal Hyperbilirubinemia

**DOI:** 10.1155/2022/5379369

**Published:** 2022-10-11

**Authors:** Zhong Chen, Qi He, Wenxing Li, Juan Liang, Tingting Zhu, Jun Tang

**Affiliations:** ^1^Department of Pediatrics, West China Second University Hospital, Sichuan University, Chengdu 610000, China; ^2^Key Laboratory of Birth Defects and Related Diseases of Women and Children, Ministry of Education, Sichuan University, Chengdu 610000, China

## Abstract

Amplitude-integrated electroencephalography (aEEG) is an effective and simple means of continuous EEG monitoring beside the neonatal bed, which can be used to predict the early brain injury and prognosis evaluation of neonatal hyperbilirubinemia. This paper summarized 11 randomized controlled studies to meta-analyze the value of aEEG in evaluating neonatal hyperbilirubinemia and acute bilirubin encephalopathy. Through the literature search of health and interest science engineering and computer in the medical databases such as Wanfang Medicine and PubMed database, the medical information literature of aEEG to evaluate the clinical value in neonatal severe hyperbilirubinemia is used, and RevMan 5.2 software is selected for metadecomposition. The experimental results show that their serum total bilirubin is significantly higher than that of normal newborns, and with the aggravation of the condition, the serum expression is higher and higher. aEEG can effectively enhance the detection rate of such sufferers and help sufferers to receive therapy as soon as possible to ensure the prognosis of children.

## 1. Introduction

Hyperbilirubinemia is one of many neonatal disorders, and the diagnosis of current neonatal hyperbilirubinemia is mainly dependent on laboratory tests, such as total bilirubin standards. Some studies have shown that elevated total bilirubin standards are an independent risk factor for developing bilirubin encephalopathy of hyperbilirubinemia in newborns, so early diagnosis and early intervention of hyperbilirubinemia in newborns are particularly critical to improving the prognosis of hyperbilirubinemia in newborns [1, 2]. In the neonatal period, the body coagulation system is still in the perfect stage, and the coagulation system is in a state of low activity. In general, spontaneous bleeding is not caused when the coagulation system is cooperating with each other. However, if the coagulation disorder is caused during the period, it may induce diseases related to abnormal coagulation function. Because the neonatal blood-brain barrier is not mature, uncombined bilirubin is easy to cross the blood-brain barrier, leading to brain injury and acute bilirubin encephalopathy(ABE). Its fatality rate is high and may cause neurological adverse neurological sequelae, such as hearing impairment, epilepsy, and cerebral paralysis. Because early brain injury has no specific clinical manifestations, it is easy to miss diagnosis [3, 4]. If it can be detected early and treated with timely intervention, neurotoxic damage can be reversed in an early stage.

Amplitude-integrated electroencephalography (aEEG) is an effective and simple means of continuous EEG monitoring beside the neonatal bed, which can be used to predict the early brain injury and prognosis evaluation of neonatal hyperbilirubinemia. At present, the main tests commonly used in the clinical evaluation of bilirubin in brain injury are brainstem auditory evoked potential(BAEP) and cranial magnetic resonance imaging(MRI), but MRI and BAEP tests still have some limitations [5]. This examination retrieved and pooled 11 randomized controlled studies and analyzed the evaluation value of aEEG for neonatal hyperbilirubinemia and acute bilirubin encephalopathy, laying the foundation for advances in medical technology.

The rest of this paper is organized as follows: Section 2 discusses related work, followed by literature information and selection criteria designed in Section 3. Section 4 shows the experimental results and analysis, and Section 5 summarizes the paper and gives a future perspective on the work.

## 2. Related Work

Hyperbilirubinemia is caused by subjoined bilirubin production, reduced metabolism, and extensive accumulation of bilirubin in the body. The most direct clinical manifestation is jaundice, and newborns are the main set of hyperbilirubinemia. Hyperbilirubinemia is mainly divided into the physiological and pathological kinds. Many neonatal hyperbilirubinemia can be normal, but some neonatal hyperbilirubinemia, especially with pathological hyperbilirubinemia neonates, if not timely intervened, will directly induce bilirubin encephalopathy and damage neonatal hearing and nervous system. Therefore, the early diagnosis and intervention of neonatal hyperbilirubinemia are very important for neonatal development. Excessive bilirubin standards may affect brain damage in children and even develop ABE. In addition, ABE has a high disability rate, which is also a current clinical concern [6]. In other countries, its incidence rate has been substantially reduced. However, in China, because some areas for the screening of newborn bilirubin are not perfect, the occurrence of the ailment is not uncommon and even shows a recovery trend. Some children with ABE will have different degrees of neurological sequelae, such as auditory impairment, eye movement disorders, and other manifestations, which will have a serious impact on the growth and development and quality of life of children. Therefore, seeking appropriate clinical tests for early detection and early diagnosis is the key to reducing sequelae and even lethality [7].

aEEG is a widely used mapping form by filtering and compressing an ordinary electroencephalogram and recording it with brain function monitoring atlas. The main working principle is as follows: aEEG is a simple single-channel electroencephalogram. The frequency of the signal of the double parietal electrode can be monitored, amplified, and filtered to form the change rule of EEG activity in a period of time so as to show the degree of nerve damage in the brain in the form of compressed integral amplitude [8]. The studies combined found that serum bilirubin standards were significantly higher in newborns with bilirubinemia than in the normal set. Serum bilirubin standards were significantly higher in neonates with severe bilirubinemia than in the mild set. The detection rate of aEEG in newborns with bilirubinemia was considerably high. The detection rate of aEEG in newborns with severe bilirubinemia was notoriously high. The disparity was more extensive (*P* < 0.05). aEEG has the following advantages: simple, easy to identify, not susceptible to drugs, bedside, continuous monitoring, etc. It has a high predictive value for brain injury and prognosis. As a method for monitoring brain function at the bedside, due to aEEG's simple operation and its noninvasive nature, the original EEG can be displayed synchronously and not affected by low voltage, which can more intuitively reflect the background changes of brain activity [9]. Moreover, the monitoring results are simple and easy in interpretation and decomposition, and they are more suitable for bedside monitoring of newborns with high-risk factors [10]. In addition, some studies have shown that aEEG has both safety and clinical feasibility, with almost no adverse events occurring, further indicating that aEEG has a high monitoring safety profile [11]. It has been shown that aEEG can be used in the early diagnosis of ABE and that the occurrence of brain injury in hyperbilirubinemia is positively associated with the abnormal degree of aEEG. The results also showed the high specificity and sensitivity of aEEG in the diagnosis of early brain injury in children with hyperbilirubinemia [12]. Through aEEG monitoring of high-risk children with nerve injury, some studies have found that aEEG appears when obvious central nervous system damage occurs, especially in children with severe injury, aEEG has a specific abnormal map [13, 14].

This study lacks support from English literature, which may lead to data bias. In this paper, aEEG is mainly used to evaluate the treatment of hyperbilirubinemia. In subsequent studies, relevant indicators can be added for systematic decomposition, and the test design and verification decomposition can be further strengthened on the basis of expanding the number of sample literature works.

## 3. Literature Information and Selection Criteria

### 3.1. Literature Information

#### 3.1.1. Examination Type

The examination and experiment type is randomized controlled trials (RCTs).

#### 3.1.2. Literature Search

Retrieving relevant clinical contrast experiments in literature databases, the examination directions are based on the evaluation of aEEG and serum bilirubin expression in severe neonatal hyperbilirubinemia. The literature search time is set to be from January 2013 to May 2022. Keywords searched are as follows: integrating hyperbilirubinemia, newborn, aEEG, abnormal rate, serum bilirubin standard, hyperbilirubinemia, neonatal, aEEG, abnormal rate, serum bilirubin standard, brainstem auditory evoked potential, and others.

### 3.2. Literature Selection Criteria

#### 3.2.1. Inclusion Criteria

The inclusion criteria are as follows:

1. The included documents are published after 2013, which is in line with the examination direction
2. The setting method is random setting
3. Comparative examination with aEEG and routine examination, respectively
4. The examination passes the examination and approval of the relevant medical institutions
5. The follow-up rate is <20%, and data integrity is high
6. A series of obvious errors in clinical laboratory indicators, including errors in aEEG, abnormal rates, and serum bilirubin standard observation indicators, are set for this examination.Q10: The sentence “A series of obvious … in this examination” is grammatically unclear. Please rephrase the sentence for clarity. Author Reply: change it to “A series of obvious errors in clinical laboratory indicators, including errors in aEEG, abnormal rate and serum bilirubin standard observation indicators set for this examination.”

#### 3.2.2. Exclusion Criteria

The exclusion criteria are as follows:

1. Poor content logic and repeated serious literature
2. Clinical experiment operation errors, incomplete data, and incomplete literature need to be excluded
3. Basic experiments such as cells and animals need to exclude studies
4. Literature inconsistent with the examination direction of this examination needs to be excluded
5. The article is the review, meta-analysis, case report, and conference summary
6. Sufferers with serious hematological ailments
7. The rate of loss to follow-up due to withdrawal or interruption of follow-up during follow-up is more than 20%

### 3.3. Examination Outcome Measures

The observed result indicators of this examination include the detection rate and the serum bilirubin standard.

### 3.4. Quality Evaluation

The modified Jadad scale is scored from 1 to 7 points, and the literature quality is evaluated using this scale, 3 as the low-quality literature and otherwise as the high-quality literature.

### 3.5. Statistical Therapy

Using RevMan5.2 statistical software, the count data are analyzed by RR as a representation, decomposition statistics are expressed as SMD, and the effect size is expressed as 95% CI. When heterogeneity is *P* < 0.1, the 50% are decomposed by the random effect model, and the rest are decomposed by the fixed model, and the difference is statistically significant.

## 4. Experimental Results

### 4.1. Literature Search Results and Characteristics of the Included Examination

Figure 1 shows the document selection flowchart.  Table 1 shows the literature inclusion information and quality. In Table 1, ① represents serum bilirubin standard (bilirubinemia), ② represents serum bilirubin standard (severe bilirubinemia), ③ represents the diagnosis rate of bilirubinemia, and ④ represents diagnosis of the severe bilirubinemia rate. As shown in Figure 1 and Table 1, a total of 11 documents conforming to the examination direction and keywords are selected after the search of the Chinese-British literature database, including 5 in English, 6 in Chinese, 3 in low-quality documents, and 8 in high-quality documents.

### 4.2. Results of the Literature Bias Decomposition

Figure 2 shows the literature bias decomposition.  Figure 3 shows the bias decomposition of the literature. It can be seen from Figures 2 and3 that the 13 included documents give detailed explanations and the methods are correct. The results of publication bias assessment show a low risk of bias in the included studies.

### 4.3. Metadecomposition Results

#### 4.3.1. Serum Bilirubin Standards' Expression in Bilirubinemic Neonates

Five references are included.  Figure 4 shows the forest plot of the expression of serum bilirubin standards in neonates with bilirubinemia.  Figure 5 shows the funnel plot of the expression of serum bilirubin standards in neonates with bilirubinemia. Through the above experimental results, it can be observed that I^2^ = 100%, *P* < 0.00001, which indicates heterogeneity among the included literature, so the random-effect model is used for decomposition. The studies found that the serum bilirubin standard is significantly higher than the normal set, with an extensive disparity (*P* < 0.05). The serum bilirubin standard can be considered as a basis for examining bilirubinemia-related ailments.

#### 4.3.2. Serum Bilirubin Standard Expression in Neonates with Severe Bilirubinemia

Figure 6 shows the forest plot of the expression of serum bilirubin standards in neonates with severe bilirubinemia.  Figure 7 shows the funnel plot of the expression of serum bilirubin standards in neonates with severe bilirubinemia. It can be seen from Figures 6 and7 that five references are included, and the heterogeneity test results show I^2^ = 98%, *P* < 0.00001, indicating heterogeneity among the included literature, so the random-effect model is used for decomposition. The studies find that the serum bilirubin standard in newborns with severe bilirubinemia showed significant difference compared to the mild set (*P* < 0.05), and the serum bilirubin standard can be considered as the basis for bilirubinemia-related ailment severity.

#### 4.3.3. Diagnosis Rate of aEEG in Neonates with Bilirubinemia

Figure 8 shows the forest plot of aEEG for the diagnosis rate of neonatal bilirubinemia.  Figure 9 shows the funnel plot of aEEG for the diagnosis rate of neonatal bilirubinemia. It can be seen from Figures 8 and9 that six references are included, and the heterogeneity test results show *I*^*2*^ = 40%, *P*=0.14, indicating that there is no heterogeneity between the included literature, so the fixed-effect model for decomposition is used. The combined studies find that contrast with routine examination, aEEG for the bilirubinemia newborn detection rate is significantly high, the disparity is extensive (*P* < 0.05), and aEEG can be considered as a means of detection for neonates with bilirubinemia.

#### 4.3.4. aEEG on the Diagnosis Rate of Newborns with Severe Bilirubinemia

Figure 10 shows the forest plot of aEEG for the diagnosis rate of severe bilirubinemia neonates.  Figure 11 shows the EEG funnel plot for the diagnosis rate of severe bilirubinemia in neonates. It can be seen from Figures 10 and11 that five references are included, and the heterogeneity test results show I^*2*^ = 0%, *P* = 0.79, indicating heterogeneity between the included literature, so the fixed-effect model is used for decomposition. The studies find that contrast with conventional examination, aEEG for the severe bilirubinemia newborn detection rate is significantly high (*P* < 0.05), the disparity is extensive, and aEEG for severe serum bilirubin standard is high and can be used as a severe bilirubinemia examination method.

### 4.4. Sensitivity Decomposition

After the sensitivity decomposition of the 13 included documents, the results after excluding and combining the examination data show that the results of each index show no extensive change, indicating that the heterogeneity among the 13 documents included in this examination is relatively small, so it has high reference value.

## 5. Conclusion

Hyperbilirubinemia is one of many neonatal disorders. For newborns with hyperbilirubinemia, their serum total bilirubin is significantly higher than that of normal newborns, and with the aggravation of the condition, the serum expression is high. aEEG can effectively enhance the detection rate of such sufferers and help sufferers to receive therapy as soon as possible to ensure the prognosis of children.

## Figures and Tables

**Figure 1:** Document selection flowchart.

**Figure 2:** Literature bias decomposition.

**Figure 3:** Bias decomposition of the literature.

**Figure 4:** Forest plot of the expression of serum bilirubin standards in neonates with bilirubinemia.

**Figure 5:** Funnel plot of the expression of serum bilirubin standards in neonates with bilirubinemia.

**Figure 6:** Forest plot of the expression of serum bilirubin standards in neonates with severe bilirubinemia.

**Figure 7:** Funnel plot of the expression of serum bilirubin standards in neonates with severe bilirubinemia.

**Figure 8:** Forest plot of aEEG for the diagnosis rate of neonatal bilirubinemia.

**Figure 9:** Funnel plot of aEEG for the diagnosis rate of neonatal bilirubinemia.

**Figure 10:** Forest plot of aEEG for the diagnosis rate of severe bilirubinemia neonates.

**Figure 11:** EEG funnel plot for the diagnosis rate of severe bilirubinemia in neonates.

**Table 1:** Literature inclusion information and quality.

First author	Year of publication	Sample capacity	Outcome indicators	Quality of the literature
Ahmadpour [15]	2018	40/30	①	4
Zhang [16]	2020	75/75	①②	4
Kumar [17]	2020	35/35	①	6
Dani [18]	2019	37/37	②	4
Tang [19]	2021	100/100	②	6
Jiang [20]	2020	40/40	①②③④	5
Chen [21]	2016	21/21	③	6
Shen [22]	2021	66/100	③④	5
Yang [23]	2020	66/66	②③④	2
Yao [24]	2017	77/70	③④	6
Wu [25]	2017	55/55	①③④	4

## Data Availability

The simulation experiment data used to support the findings of this study are available from the corresponding author upon request.
